The article "Mirtazapine prevents cell activation, inflammation, and oxidative stress against isoflurane exposure in microglia" was retracted in 2024. Reasons: original data or images not available; unreliable results or conclusions; concerns about the data; concerns about the results or conclusions.

# Mirtazapine prevents cell activation, inflammation, and oxidative stress against isoflurane exposure in microglia

**DOI:** 10.1080/21655979.2021.2009971

**Published:** 2021-12-29

**Authors:** Qi Wang, Meina Ma, Hong Yu, Hongmei Yu, Shuai Zhang, Rui Li

**Affiliations:** Department of Anesthesiology, Cangzhou Central Hospital, Cangzhou, Hebei, China

**Keywords:** Mirtazapine, isoflurane, cognitive dysfunction, microglia activation, neuroinflammation, oxidative stress

## Abstract

Mirtazapine is an antidepressant drug that has been proven to possess a cognitive enhancer efficiency. In this study, we evaluated the potential protective effects of mirtazapine on BV2 microglia in response to isoflurane exposure. Our results show that mirtazapine attenuated isoflurane-induced expression of microglia-specific protein Iba1 in BV2 microglia. Mirtazapine prevented isoflurane-induced production of the pro-inflammatory factors interleukin (IL)-1β and IL-18 by inhibiting the activation of the nod-like receptor family protein 3 (NLRP3) inflammasome in BV2 microglia. The increased reactive oxygen species (ROS) production and elevated expression level of NADPH oxidase 4 (NOX4) in isoflurane-induced BV2 microglia were mitigated by mirtazapine. Isoflurane exposure reduced triggering receptor expressed on myeloid cells 2 (TREM2) expression in BV2 microglia, which was restored by mirtazapine. Moreover, silencing of TREM2 abolished the inhibitory effects of mirtazapine on ionized calcium-binding adapter molecule 1 (Iba1) expression and inflammation in BV2 microglia. From these results, we could infer that mirtazapine exerted a protective effect on BV2 microglia against isoflurane exposure-caused microglia activation, neuroinflammation, and oxidative stress via inducing TREM2 activation. Hence, mirtazapine might be a potential intervention strategy to prevent isoflurane exposure-caused cognitive dysfunction in clinical practice.

## 1. Introduction

Isoflurane is an inhaled anesthetic widely used in clinical practice with multiple advantages like satisfactory anesthetic effects, rapid induction and recovery, ease of anesthetic depth adjustment, as well as low toxicity on circulation [1]. However, it has been reported that patients with isoflurane usage exhibit an increased postoperative cognitive dysfunction (POCD) risk, which is a common central nervous system (CNS) disorder [2]. Isoflurane-associated POCD has a significant negative impact on patients’ psychomotor functions, attention and memory, and has become a public health concern [3]. Prior studies have documented that neuroinflammation is critical in the pathogenesis of isoflurane-induced cognitive dysfunction. Microglia are the immune effector cells in the brain that play a crucial role in maintaining the homeostasis of brain tissues [4]. In response to specific stimuli, microglia are activated to secrete pro-inflammatory factors, thereby causing neuroinflammation, damage to neurons, and death [5]. Iba1 is a novel calcium-binding protein that is specifically expressed in microglia. Recently, Iba1 has been considered a biomarker of microglia activation [6]. It is conceivable that microglia activation is a considerable negative event in the development of neurocognitive disorders. The activated NLRP3 inflammasome plays a pivotal role in neurocognitive disorders by releasing IL-1β and IL-18, resulting in neuroinflammation and cell death. TREM2 is an immunomodulatory receptor exclusively expressed on immune cells, including microglia, and it regulates various cell functions such as inflammatory response. Therefore, appropriate inhibition of microglia activation can be conducive to formulating effective therapeutic strategies for associated pathological damages [7].

The article "Mirtazapine prevents cell activation, inflammation, and oxidative stress against isoflurane exposure in microglia" was retracted in 2024. Reasons: original data or images not available; unreliable results or conclusions; concerns about the data; concerns about the results or conclusions.

Mirtazapine is a well-established antidepressant drug used for relieving depression, anxiety, and sleep disturbance symptoms of patients suffering from depression [8]. In recent years, mirtazapine has been proven to possess a cognitive enhancer efficiency. It was reported to potentially improve cognitive dysfunctions in the treatment of chronic schizophrenia [9,10]. Mirtazapine has a therapeutic potency against neurodegenerative diseases, such as Parkinson’s disease and Alzheimer’s disease. Its administration causes increased motor dysfunction and facilitated utilization of dopamine in 1-methyl-4-phenyl-1,2,3,6- tetrahydropyridine (MPTP)-induced mice models [11]. Mirtazapine also improves auditory and visual hallucinations in patients with Parkinson’s disease. Cakir et al. [12] reported that mirtazapine is effective for the treatment of agitated Alzheimer’s disease patients without significant side effects and cognitive deterioration. Additionally, it has been reported to exert inhibitory effects on neuroinflammation. Based on the findings from previous studies, we speculate that mirtazapine might have a protective property against isoflurane. In this study, we aimed to investigate its beneficial effects on isoflurane-challenged BV2 microglial cells and explored the underlying mechanism.

## 2. Materials and methods

### 2.1. Cell culture and transduction

Murine BV-2 microglial cells were cultred in low glucose (5 mM) RPMI1640 medium with penicillin (100 U/ml), streptomycin (100 µg/ml), and 10% FBS. The BV-2 cells were maintained in 5% CO_2_ at 37°C. To obtain TREM2-silencing cells, BV-2 microglia were introduced with adenovirus carrying TREM2 shRNA (Ad-TREM2 shRNA), which was obtained from HanBio. (Shanghai, China). The BV2 microglia introduced with Ad-control shRNA were used as the control. Western blot analysis was applied for the determination of silence efficiency. To measure the cytotoxicity of mirtazapine in BV2 microglia, the cells were stimulated with 0, 1.5, 3, 15, 30, 150, 300 μM for 24 hours. To evaluate the protective effects of mirtazapine against isoflurane in BV-2 microglia, the cells were treated with 3% Isoflurane [13] with or without Mirtazapine (15, 30 μM) for 24 hours. Cells treated with DSMO were used for vehicle control.

The article "Mirtazapine prevents cell activation, inflammation, and oxidative stress against isoflurane exposure in microglia" was retracted in 2024. Reasons: original data or images not available; unreliable results or conclusions; concerns about the data; concerns about the results or conclusions.

### 2.2. Lactate dehydrogenase (LDH) release assay

Cell damage of BV-2 cells was examined by determining LDH release into the cell medium after incubation with mirtazapine (0, 1.5, 3, 15, 30, 150, 300 μM) for 24 h, using an LDH assay kit (Pierce, Rockford, IL, USA). Absorbance was read at 490 nm on a Flexstation 3 plate reader [14].

### 2.3. Reactive oxygen species (ROS) generation detection

The production of ROS by BV-2 cells was assessed using 2ʹ,7ʹ-Dichlorofluorescin diacetate (DCFH-DA), which is a fluorescent probe. Following the indicated treatment, DCFH-DA (10 µM) was added to the cells and incubated for 25 min. Fluorescent images were captured with a fluorescent microscope (Olympus, Tokyo, Japan). The fluorescent intensity of ROS was quantified using the Image J software [15].

### 2.4. Real-time quantitative reverse transcription PCR (qRT-PCR)

Following treatment, the mRNA levels of NOX-4,Iba1, NLRP3, IL-1β, IL-18, and TREM2 were detected by qRT-PCR as described previously [16] with a High Capacity cDNA Archive Kit and SYBR Green Master mix (Applied Biosystems, Foster City, CA, USA). The relative expressions of target genes were determined by the 2^−ΔΔCq^ method relative to an internal control, GAPDH. The following primers were used in this study: IL-1β, F: 5ʹ-AGGAGAACCAAGCAACGACA-3ʹ,R:5ʹ-CTCTGCTTGTGAGGTGCTGA-3ʹ; IL-18, F: 5ʹ-ACCAAGTTCTCTTCGTTGAC-3ʹ, R: 5ʹ-CTTCACAGAG AGGGTCACAG-3ʹ; Iba1, F: 5ʹ-ATGAGCCAAAGCAGGGATTT-3ʹ, R: 5ʹ-TTG GGATCATCGAGGAATTG-3ʹ; NLRP3, F: 5ʹ-ATTACCCGCCCGAGAAAGG −3ʹ, R: 5ʹ-CATGAGTGTGGCTAGATCCAAG −3ʹ; TREM2, F: 5ʹ- CTGGAACCGTCACCATCACTC-3ʹ, R: 5ʹ-CGAAACTCGATGACTCCTCGG −3ʹ; Nox-4, F: 5ʹ-TGCCT GCTCATTTGGCTGT-3ʹ, R: 5ʹ- CCGGCACATAGGTAAAAGGATG −3ʹ; GAPDH, F: 5ʹ-TGACCTCAACTACATGGTCTACA-3ʹ, R: 5ʹ-CTTCCCATTCTCGGCCTTG-3ʹ.

### 2.5. Western blot

Total proteins of BV-2 cells were prepared for the determination of the protein levels of NOX-4, Iba1, NLRP3 and TREM2 with Western blot analysis as previously described [17]. The primary antibodies in this study include anti-NOX-4 (1:2000, #ab133303, Abcam, USA), anti-Iba1 (1:2000, #ab178846, Abcam, USA), anti-NLRP3 (1:2000, #ab263899, Abcam, USA), anti-TREM2 (1: 1000, #ab209814 Abcam, USA) and anti-β-actin (1:5000, #ab179467, Abcam, USA), and the secondary antibodies (1:2000 #ab150117 Abcam Cambridge, MA, USA). Upon completion of the Western blot assay, the blots were analyzed using NIH Image J software. The following antibodies were used in this study: anti-NOX-4 (#ab133303, Abcam, USA), anti-Iba1 (#ab178846 Abcam, USA), anti-NLRP3 (#ab263899, Abcam, USA), anti-TREM2 (#ab209814, Abcam, USA), anti-β-actin (#ab179467, Abcam, USA) and the secondary antibodies (#ab150117, Abcam, USA).

The article "Mirtazapine prevents cell activation, inflammation, and oxidative stress against isoflurane exposure in microglia" was retracted in 2024. Reasons: original data or images not available; unreliable results or conclusions; concerns about the data; concerns about the results or conclusions.

### 2.6. Enzyme-linked immunosorbent assay (ELISA)

IL-1β and IL-18 levels from the BV-2-conditioned medium were measured using ELISA kits from Biolegend (San Diego, CA, USA) based on the protocol provided by the manufacturer. Absorbance was detected at 450 nm using Flexstation 3 plate reader [18].

### 2.7. Data analysis

Data were analyzed for statistical comparisons using GraphPad Prism (version 8.01) with the analysis of variance (ANOVA) method. Data were represented as the mean value +/− SEM. *p*< 0.05 was used as a threshold to indicate statistically significant differences.

## 3. Results

Firstly, we tested the cytotoxicity of mirtazapine in BV2 cells. Secondly, we measured the expression of Iba1, which is an important biomarker of microglia activation. Then, we investigated the effect of mirtazapine on NLRP3 inflammasome activation, which is responsible for the expressions of IL-1β and IL-18. Furthermore, we examined the levels of ROS and NOX-4, to clarify the potential benefits of mirtazapine against oxidative stress. Lastly, we investigated the involvement of TREM2 in isoflurane-challenged BV2 cells.

### 3.1. The cytotoxicity of mirtazapine in BV2 microglia

BV2 microglia were stimulated with 0, 1.5, 3, 15, 30, 150, and 300 μM of mirtazapine for 24 h. The cytotoxicity of mirtazapine (structure shown in Figure 1(a)) in BV2 microglia was analyzed using LDH release assay as shown in Figure 1(b). No significant changes were observed in BV2 microglia treated with 1.5, 3, 15, and 30 μM mirtazapine, while obviously increased LDH release levels were noted in BV2 microglia treated with 150 and 300 μM mirtazapine.

**Figure 1.** The cytotoxicity of mirtazapine in BV2 microglia. Cells were stimulated with 0, 1.5, 3, 15, 30, 150, 300 μM for 24 hours. (a) Molecular structure of Mirtazapine; (b) Cytotoxicity of BV2 microglia was measured using LDH release assay (^***^P < 0.05, 0.01 vs. Vehicle group, n = 5).

### 3.2. Mirtazapine reduced isoflurane-induced expression of Iba1 in BV2 microglia

In qRT-PCR analysis (Figure 2(a)), the mRNA level of the microglia-specific protein Iba1 was proven to be upregulated by 2.7-fold in isoflurane-induced BV2 microglia. However, mirtazapine (15, 30 μM) prevented this upregulation of Iba1 mRNA. Similarly, in Western blot analysis (Figure 2(b)), isoflurane effectively induced an increase in the protein level of Iba1 in BV2 microglia with a 2.5-fold change, which would be reversed by mirtazapine (15, 30 μM).

The article "Mirtazapine prevents cell activation, inflammation, and oxidative stress against isoflurane exposure in microglia" was retracted in 2024. Reasons: original data or images not available; unreliable results or conclusions; concerns about the data; concerns about the results or conclusions.

**Figure 2.** Mirtazapine inhibited isoflurane-induced expression of Iba1 in BV2 microglial cells. Cells were stimulated with 3% isoflurane with or without mirtazapine (15, 30 μM) for 24 hours. (a) mRNA level of Iba1; (b) Protein level of Iba1 (***P < 0.005 vs. vehicle group; ^#,^^##^P < 0.05, 0.01 vs. isoflurane group, n = 6).

### 3.3. Mirtazapine suppressed isoflurane-induced activation of the NLRP3 inflammasome in BV2 microglia

In order to investigate the effect of mirtazapine on isoflurane-induced activation of the NLRP3 inflammasome, cells were stimulated with 3% Isoflurane with or without Mirtazapine (15, 30 μM) for 24 hours. Further analysis of the NLRP3 inflammasome showed that its mRNA level was significantly increased by 3.3-fold in isoflurane-induced BV2 microglia, while 30.3% and 48.5% reduction were respectively observed in BV2 microglia treated with 15 or 30 μM mirtazapine (Figure 3(a)). We next found a 2.7-fold increase in the protein level of NLRP3 in isoflurane-induced BV2 microglia. Mirtazapine (15, 30 μM) treatment reduced the NLRP3 protein level in BV2 microglia against isoflurane-caused induction (Figure 3(b)).

**Figure 3.** Mirtazapine suppressed isoflurane-induced activation of NLRP3 inflammasome in BV2 microglial cells. (a) mRNA level of NLRP3; (b) Protein level of NLRP3 (***P < 0.005 vs. vehicle group; ^#,^^##^P < 0.05, 0.01 vs. isoflurane group, n = 6).

### 3.4. Mirtazapine inhibited the secretions of IL-1β and IL-18 in BV2 microglia

We showed that the mRNA levels of IL-1β and IL-18 in BV2 microglia were dramatically increased by 3.7- and 3.2-fold, respectively, after stimulation with 3% isoflurane. Mirtazapine (15, 30 μM)-treated BV2 microglia displayed a significant decrease in the mRNA levels of IL-1β and IL-18 (Figure 4(a)). As expected, ELISA provided consistent results in the inhibitory effects of mirtazapine (15, 30 μM) on the secretions of IL-1β and IL-18 in 3% isoflurane-stimulated BV2 microglia (Figure 4(b)).

**Figure 4.** Mirtazapine inhibited the secretions of IL-1β and IL-18 in BV2 microglial cells. (a) mRNA level of IL-1β and IL-18; (b) Secretions of IL-1β and IL-18 (***P < 0.005 vs. vehicle group; ^#,^^##^P < 0.05, 0.01 vs. isoflurane group, n = 5).

### 3.5. Mirtazapine attenuated isoflurane-induced oxidative stress in BV2 microglia

Cells stimulated with 3% isoflurane showed a remarkable increase (2.8-fold) in the intracellular ROS level, as seen from Figure 5(a). In the presence of mirtazapine (15, 30 μM), the increased intracellular ROS level was decreased by 32.1% and 50.0%, respectively. Next, we also observed that 3% isoflurane induction caused significant 3.4-fold and 3.1-fold increases in mRNA and protein levels of NOX-4 in BV2 microglia (Figure 5b,figure 5c). However, these changes were dose-responsively mitigated by mirtazapine (15, 30 μM).

The article "Mirtazapine prevents cell activation, inflammation, and oxidative stress against isoflurane exposure in microglia" was retracted in 2024. Reasons: original data or images not available; unreliable results or conclusions; concerns about the data; concerns about the results or conclusions.

**Figure 5.** Mirtazapine attenuated isoflurane-induced oxidative stress in BV2 microglial cells. Cells were stimulated with 3% isoflurane with or without mirtazapine (15, 30 μM) for 24 hours. (a) Intracellular ROS; Scale bar, 100 μm; (b) mRNA level of NOX-4; (c) Protein level of NOX-4 (***P < 0.005 vs. vehicle group; ^#,^^##^P < 0.05, 0.01 vs. isoflurane group, n = 5).

### 3.6. Mirtazapine restored isoflurane-induced reduction of TREM2 in BV2 microglia

Subsequently, we found that 3% isoflurane induced a significant reduction (0.53-fold) in the mRNA level of TREM2 (Figure 6(a)). This influence of 3% isoflurane on the mRNA level of TREM2 was attenuated by mirtazapine (15, 30 μM). Furthermore, as shown in Figures 6(b), 3% isoflurane-induced decrease (0.57-fold) in the protein level of TREM2 was also reversed by mirtazapine (15, 30 μM).

**Figure 6.** Mirtazapine restored isoflurane-induced reduction of TREM2 in BV2 microglial cells. (a) mRNA level of TREM2; (b) Protein level of TREM2 (***P < 0.005 vs. vehicle group; ^#,^^##^P < 0.05, 0.01 vs. isoflurane group, n = 6).

### 3.7. Silencing of TREM2 abolished the protective effects of mirtazapine against isoflurane in BV2 microglia

To clarify the involvement of TREM2, its expression was knocked down by transduction with Ad-TREM2 shRNA. We observed that this induced a 48% reduction in TREM2 protein expression (Figure 7(a)). Interestingly, the inhibitory effects of mirtazapine in the expression of the NLRP3 protein were abolished by mirtazapine (Figure 7(b)). Correspondingly, the deceased secretion levels of IL-1β and IL-18 in mirtazapine (30 μM)-treated BV2 microglia were elevated after transduction with Ad-TREM2 shRNA (Figure 7(c)).

**Figure 7.** Silencing of TREM2 abolished the protective effects of mirtazapine against isoflurane in BV2 microglial cells. Cells were transduced with Ad-TREM2 shRNA, followed by stimulation with 3% isoflurane or mirtazapine (30 μM) for 24 hours. (a) Western blot results of TREM2; (b) Protein level of NLRP3; (c) Secretions of IL-1β and IL-18 (***P < 0.005 vs. vehicle group; ^#,^^##^P < 0.005 vs. isoflurane group; ^#,^^##^P < 0.005 vs. isoflurane+mirtazapine group, n = 5).

The article "Mirtazapine prevents cell activation, inflammation, and oxidative stress against isoflurane exposure in microglia" was retracted in 2024. Reasons: original data or images not available; unreliable results or conclusions; concerns about the data; concerns about the results or conclusions.

### 3.8. Silencing of TREM2 abolished the inhibitory effects of mirtazapine on Iba1 expression in BV2 microglia

In BV2 microglia introduced with Ad-TREM2 shRNA, the mRNA level of Iba1 in the mirtazapine (30 μM)-treated group was elevated to the same level as that in 3% isoflurane-induced BV2 microglia (Figure 8(a)). A similar effect from the silencing of TREM2 was observed on the protein level of Iba1 (Figure 8(b)).

**Figure 8.** Silencing of TREM2 abolished the inhibitory effects of mirtazapine in Iba1 expression in BV2 microglial cells. Cells were transduced with Ad-TREM2 shRNA, followed by stimulation with 3% isoflurane or mirtazapine (30 μM) for 24 hours. (a) mRNA level of Iba1; (b) Protein level of Iba1 (***P < 0.005 vs. vehicle group; ^#,^^##^P < 0.005 vs. isoflurane group; ^#,^^##^P < 0.005 vs. isoflurane+mirtazapine group, n = 6).

## 4. Discussion

Recent researches have demonstrated that microglia serve diverse functions in the CNS during aging, health, and neurodegenerative disorders [19]. The role of microglia in the CNS can be neurotoxic or neuroprotective, depending on the activation status. Pro-inflammatory cytokines from damaged cells, or specific stimuli, have the capacity to activate the resting microglia. The activation of microglia thus induces the expressions of pro-inflammatory factors such as IL-1β, IL-18, TNF-α, and nitric oxide (NO), which have detrimental effects on neurons [20]. Based on previous cellular and animal experiments, isoflurane exposure induces the activation of microglia and exerts detrimental effects [21]. In a POCD mice model, isoflurane anesthesia causes impaired spatial learning memory, which is associated with microglia activation accompanied by the increased expressions of IL-1β, TNF-α, and IFN-γ [22]. Isoflurane induces neuronal apoptosis and neuroinflammation in rats, switches microglia polarization, and increases pro-inflammatory factors IL-1β, IL-6, IL-18, TNF-α, and iNOS expressions in BV2 cells [21]. Therefore, we attempted to investigate the effect of mirtazapine on Isoflurane-mediated BV2 microglia activation. In our experiments, we tested the cytotoxicity of mirtazapine in BV2 microglia. The results show that when the concentration of mirtazapine is lower than 30 μM, it has no significant impact on the viability of BV-2 cells, suggesting treatment with lower concentrations of mirtazapine has no side effect on the biology of BV-2 cells.

It has been identified that Iba1 expression is upregulated in activated microglia [23,24]. Here, we found that mirtazapine attenuated the isoflurane-induced increased expression of Iba1 in BV2 microglia. NLRP3 is a key component of the inflammasome in microglia, and its activation triggers the cleavage of pro‐IL‐1β and pro‐IL‐18 to their active forms by Caspase-1, after which pyroptosis ensues, eventually resulting in cell death [25]. We found that mirtazapine inhibited the activation of the NLRP3 inflammasome in isoflurane-induced BV2 microglia. The isoflurane-induced production of the pro-inflammatory factors IL-1β and IL-18 was prevented by mirtazapine. In addition to the overproduction of pro-inflammatory factors, activated microglia also release excessive ROS that cause oxidative damage in neurons, another mechanism of microglia-mediated neurotoxicity together with neuroinflammation [26,27]. For numerous neurotoxic stimuli, NADPH oxidase (NOX) is the primary source of ROS. NOX isoforms, NOX2, and NOX4 are activated and play a key role in microglial ROS production in response to neurotoxic stimuli [28]. Our results show that the increased ROS production and elevated expression level of NOX4 in isoflurane-induced BV2 microglia were mitigated by mirtazapine. These findings suggest that mirtazapine protected BV2 cells from isoflurane-induced microglia activation, neuroinflammation, and oxidative stress.

The article "Mirtazapine prevents cell activation, inflammation, and oxidative stress against isoflurane exposure in microglia" was retracted in 2024. Reasons: original data or images not available; unreliable results or conclusions; concerns about the data; concerns about the results or conclusions.

TREM2 signaling is involved in cell activation, survival, inflammation, regulation, and phagocytosis [29]. Its expression is dramatically altered in response to inflammatory stimuli and injuries. *In vitro*, the application of pro-inflammatory molecules such as TNF-α, IL-1β, ROS, and IFN-γ causes a decrease in TREM2 expression [30]. Previous studies have found that the dysregulation of TREM2 is strongly correlated to neuropathology [31]. It is reported that TREM2 regulates microglial functions and acts as a marker of microglial activation. TREM2 knock-out (TREM2^−/−^) microglia were found to exhibit reduced clearance of dying cells [32]. TREM2^−/−^ mice have decreased microglial survival and impaired microglial response [33]. In this study, we clarified the effects of mirtazapine on TREM2 expression in isoflurane-challenged BV-2 microglia. Our results prove that isoflurane exposure caused reduced TREM2 expression in BV2 microglia, which was restored by mirtazapine. Moreover, silencing of TREM2 abolished the inhibitory effects of mirtazapine on Iba1 expression and inflammation in BV2 microglia. The main limitation of the current study is that we only examined the protective effects of mirtazapine against isoflurane-induced microglia activation in an *in vitro* BV-2 model. It should be noted that the pathological mechanism of isoflurane-associated POCD is complicated and needs further elucidation. Future *in vivo* studies with animal models are necessary to verify the function of mirtazapine in isoflurane-induced microglia activation.

The article "Mirtazapine prevents cell activation, inflammation, and oxidative stress against isoflurane exposure in microglia" was retracted in 2024. Reasons: original data or images not available; unreliable results or conclusions; concerns about the data; concerns about the results or conclusions.

## 5. Conclusion

In summary, from these results, we can infer that mirtazapine exerted a protective effect on BV2 microglia against isoflurane exposure-caused microglia activation, neuroinflammation, and oxidative stress via inducing TREM2 activation. Hence, mirtazapine might be a potential intervention strategy to prevent isoflurane exposure-caused cognitive dysfunction in clinical practice.

## Data Availability

Requests for data and materials should be addressed to the corresponding author.
